The article "Ethnobotanical and Biochemical Study of Berberis lycium Royle Collected from Different Areas of Azad Jammu and Kashmir" was published in 2021. Journal: Evid Based Complement Alternat Med.

# Ethnobotanical and Biochemical Study of *Berberis lycium* Royle Collected from Different Areas of Azad Jammu and Kashmir

**DOI:** 10.1155/2021/9916305

**Published:** 2021-09-25

**Authors:** Syeda Maria Fiaz Bukhari, Ghazanfar Ali, Syed Rizwan Abbas, Zeeshan Anjum, Nasim Ahmed, Ammara Munir, Abdul Wali, Muhammad Ayub, Kafaitullah Khan, Ahmed Khames, Muneeb Muhamed Musthafa

**Affiliations:** ^1^Department of Biotechnology, University of Azad Jammu Kashmir, Muzaffarabad, Pakistan; ^2^Department of Biological Sciences, Karakoram International University, Gilgit, Pakistan; ^3^Agricultural Biotechnology Division, National Institute for Biotechnology and Genetic Engineering College, Pakistan Institute of Engineering and Applied Sciences, Faisalabad, Pakistan; ^4^Department of Biotechnology, Virtual University of Pakistan, Lahore, Pakistan; ^5^Faculty of Life Sciences &Informatics, Balochistan University of Information Technology, Engineering and Management Sciences, 87100 Quetta, Pakistan; ^6^Institute of Biochemistry, University of Balochistan, Quetta, Pakistan; ^7^Department of Microbiology, University of Balochistan, Quetta 87300, Pakistan; ^8^Department of Pharmaceutics and Industrial Pharmacy, College of Pharmacy, Taif University, P.O. Box 11099, Taif 21944, Saudi Arabia; ^9^Department of Biosystems Technology, Faculty of Technology, South Eastern University of Sri Lanka, University Park, Oluvil #32360, Sri Lanka

## Abstract

*Berberis lycium* Royle has a long history of medicinal uses to treat different diseases. It naturally grows on the mountains of Indian subcontinent. Its ethnobotanical and biochemical study from the state of Azad Jammu and Kashmir (AJ&K) was not previously explored. So, the objective of the current study was to explore the ethnobotanical and biochemical properties of the *B. lycium* Royle population of AJ&K. For this purpose, samples of *B. lycium* Royle were randomly collected from five districts of Azad Jammu and Kashmir, including thirty-five locations. Demographic features of informants such as plant part used, methods of preparation, modes of administration, conservation status, and ethnomedicinal uses were documented. It was used for treating different diseases such as diabetes, arthritis, joint pain, and stomach ulcer. This plant is very famous for providing medicinal roots, leaves, and fruits which are extensively used in many parts of the world. The biochemical analysis was conducted for total phenolic contents (TPC), chlorophyll contents, and antioxidant activity. The highest level of TPC found was 88.66 ± 1.07 *µ*g/g of gallic acid equivalent phenolic (GAE) from leaves collected from Patikka (Chanjhal), Muzaffarabad District, AJ&K. The highest total chlorophyll contents (3.75 ± 0.53 *µ*g/ml) were found in samples collected from Sathrian, Neelum District. The highest antioxidant activity with lowest IC50 value (33.26 *µ*g/ml) was obtained from the root of sample collected from Bakreyali, Muzaffarabad District, as compared with other districts. The concentration of berberine was found to be 4.76 percent in the root bark of *B. lycium* Royle, estimated by high-performance liquid chromatography (HPLC). In syrup composition, 0.95 mg/5 ml of berberine was used. Hence, it is concluded that amongst the five districts, the plant parts (stem, fruits, and root) collected from Muzaffarabad District, AJ&K, showed the highest medicinal potential due to its unique climatic conditions.

## 1. Introduction

Medicinal plants have been utilized as folk medicines for centuries, and many communities still depend on these plants for acquiring their primary health care needs [1]. In some cultures, plants are used because of their hallucinogenic character. In many parts of the world, veterinary therapeutics also use active compounds from plants [2]. Aromatic plants have high medicinal value and have long history of use as an effective and cheap source of remedy for several health disorders [3]. An ethnobotanical study showed that people get food, fodder for animals, medicine, material for building houses, crafts, tools of agriculture, and many other products such as poisons, resins, fuel, and paints from large number of less familiar plant resources which are present in nature as today's need [4, 5]. There are different techniques and protocols used to achieve ethnobotanical knowledge (qualitative or quantitative method) about specific plants and their uses as well as caste or race's feature or study of a region [5, 6]. *Berberis lycium* Royle is a high value medicinal plant with known history in folklore medicine and traditionally used to treat different human diseases [7], such as diabetes mellitus, liver disorders, abdominal problems, skin diseases, oral ulcers, kidney, conjunctivitis, piles, leprosy, jaundice, rheumatism, and bone fractures [7–9]. It has antiglycation and antidiabetic potential and is also used to treat jaundice, bone fractures, ophthalmic disorders, fever, menorrhagia, internal wounds, intestinal colic, throat pain, diarrhea, piles, and rheumatism [10]. Thus, it has acceptance among traditional medical practitioners [8]. Furthermore, it has been used either as a food [11] or as medicine [12] because of the presence of berberine, chinabine, balauchistanamine, karakoramine, palmatine, jhelumine, gilgitine, punjabine, sindamine, ascorbic acid, maleic acid, and acetic acid [13]. Berberine is one of the most abundant alkaloid in plant [14, 15]. Berberine shows significant phytotherapeutic benefits, such as antidiarrheal, antimicrobial, antitoxic, antiprotozoal, and antitrachoma activities [10, 16]. According to different studies, berberine can be extracted from *B. lycium* roots, fruits, leaves, and stem and used for the treatment of diabetes [9]. The root bark and extract are used in treating throat pain, dysentery, internal wounds, and sun blindness [7]. The root bark water extract is used against scabies, pustules, diabetes, and bone fracture [17]. The watery extract from the root is also used in wounds, gonorrhea, curative piles, unhealthy ulcers, acute conjunctive, ophthalmia (swollen and sore eyes), and jaundice [7]. Fruits and leaves are used for the treatment of diabetes and other diseases in Pakistan [18]. The whole plant is used for curing diabetes and other human illnesses [19]. The plant growth and development are dependent upon reactive oxygen species (ROS) production and signaling as ROS play key role in plant phytohormonal networks [20], which are produced during the cellular respiration. Antioxidants scavenge these ROS and synthetic antioxidants could create toxic effects, so natural antioxidants are preferred. Compounds from plants having high antioxidant effects could be a choice to develop new medicines [21]. *B. lycium* Royle is native to the Himalayan region. Its roots are rich in alkaloids (berberine, etc.) and yellowish in color and have other phytochemicals [22]. It contains Cu, Mn, Ca, K, P, vitamin A, vitamin C, and vitamin E. Ca is helpful in strengthening bones and teeth [7]. Zn and Cu are part of dietary sources involved in redox and enzymatic reactions [8]. K and Na are involved in membrane functions. Fe is the central atom of hemoglobin which helps in electron and oxygen carrier [15]. It is also attributed to prevention of cancer and atherosclerosis. Vitamin C is a cofactor of enzymes [7]. Animal and human studies showed that optimal intake of minerals such as Cu, K, Zn, Mn, and Ca decreases risk factors, including those related to cardiovascular disorders [15, 23]. The purpose of the present study was to collect ethnobotanical knowledge about *B. lycium* Royle from major growing areas of Azad Jammu and Kashmir (AJ&K) and also its total phenolic contents, chlorophyll contents, antioxidant activity, and HPLC analysis from different places and to find the best environment for its maximum medicinal potential.

## 2. Materials and Methods

The current research was carried out for ethnobotanical and biochemical study of *B. lycium* Royle from five districts of AJ&K region, i.e., Muzaffarabad, Hattian, Bagh, Poonch, and Neelum, as shown (Figure 1). The selection of these five districts is due to their major contribution to the production of *B. lycium* Royle in the region. This study was conducted from May 2014 to July 2017 by the Department of Biotechnology, University of Azad Jammu and Kashmir (UAJ&K). This region is located between 73–75° East longitude and 33–35° North latitude and covers an area of 13,297 km^2^. The altitude of the study area varies between 600 m and 6325 m and so is the varying climate of the area. The verbal consent was obtained from each informant before conducting the interview process. The ethnobotanical study was completed in four phases: (i) description/selection of study area/locations, (ii) ethnomedicinal field survey (primary data), (iii) sample collection and their biochemical analysis (total phenolic compounds, chlorophyll contents, and antioxidant activity), and (iv) statistical analysis (secondary data) and data compilation/documentation.

### 2.1. Field Survey and Data Collection

The study area was consistently visited from May 2014 to July 2017. The prime spots were selected from AJ&K region, i.e., Muzaffarabad, Hattian, Bagh, Poonch, and Neelum. Fieldwork was implemented for the conservation status of plant and plant diversity. The field work included observations, interviews, and guided field walks. During fieldwork, two methods were frequently used. The field survey aimed to gather field data and activities, such as (i) plant collection, (ii) local knowledge regarding medicinal plant, (iii) identifying related significance to plants, (iv) conservation requisites, (v) medicinal uses, (vi) mode of preparation, and (vii) diseases treated through well-planned questionnaires, interviews, and keen observations. The questionnaire and interview method helped to document indigenous folk knowledge by involving knowledgeable persons (hakims, farmers, herdsmen, etc.) The plants were collected, and their traditional uses were asked from individuals. The plant's use which is just mentioned by one or two people is also important, but their reliability ratio is lesser, and it indicates that traditional knowledge of area about plants is disappearing from the area [2]. An ethnobotanist may use qualitative or quantitative method depending on the purpose of study [24]. The ethnobotanical data were tested and matched with the existing literature and were analyzed both qualitatively and quantitatively. During fieldwork, interviews were conducted with local inhabitants. In the interview system, a questionnaire method was used to take interviews from houses, markets, or fields. The use of local languages was preferred for collecting data because it is very essential to know the real facts about local flora [25] and local peoples. During this process, local methods of collection, drying, storage, harvesting, utilization, and processing of *Berberis lycium* Royle were practiced and noted. The plants' flowering/fruiting seasons were noted, and flowers/fruits were pressed and preserved at the same time during the ethnobotanical study of plant. All the samples were recorded in three replicates. One-way ANOVA (*P* < 0.05) was performed for statistical analysis of the data.

### 2.2. Identification of Plant

The collected plant species was identified by Dr. Tariq, Department of Botany, University of Azad Jammu & Kashmir. The accession number of plants is AKASH 000601, and voucher number is SMF-01. Biochemical analysis was also conducted on these samples collected from five districts of AJ&K (Figure 1). The biochemical analysis was carried out on the samples of *B. lycium* Royle for the estimation of phenolic contents, chlorophyll contents, and antioxidant activity.

### 2.3. Estimation of Total Phenolic Contents (TPC)

The total phenolic contents were determined by adding 0.5 mL of the plant extract to 2.5 mL of Folin–Ciocâlteu's phenol reagent (10% *v*/*v*) and 2 mL of NaHCO3 (7.5% *w*/*v* in water). The reaction mixture was incubated at 45°C for 40 min, and the absorbance was measured at 765 nm using a spectrophotometer. Distilled water was used as a standard phenol [26]. Different concentrations of gallic acid were measured to find the linear regression using the following equation:

(1) $$\begin{array}{c} y=0.0012x+0.0396R^{2}=0.9991. \end{array}$$

### 2.4. Estimation of Chlorophyll

The leaf samples (1 cm^2^) of each ecotype were taken with 5 ml ethanol in a test tube. The test tubes with samples were kept overnight to extract the chlorophyll contents. The chlorophyll extraction was measured spectrophotometrically at 646.6 nm and 663.6 nm. The values were calculated using the formula [27].

### 2.5. Antioxidant Activity by 2,2-Diphenyl-1-picrylhydrazyl (DPPH) Radical Scavenging

The antioxidant activities of the plant extract were measured by using the stable DPPH radical according to the method of [11]. 0.25 mM solution of DPPH radical (0.5 ml) was added to the sample solution in ethanol (1 ml) at different concentrations of aqueous extract of *B. lycium* Royle. The mixture was shaken vigorously and left to stand for 30 minutes in the dark, and the absorbance was measured at 517 nm. The capacity to scavenge the DPPH radical was calculated using the following equation: percentage scavenging = [(*Ao* − *As*)/*Ao*)] ^∗^ 100, where *Ao* is the absorbance of the control reaction and *As* is the absorbance of the sample itself. IC50 was calculated after plotting data and getting the linearity correlation equation.

### 2.6. Preparation of Syrup Formation

The root bark of *B. lycium* Royle was selected from Muzaffarabad District (Patkai) The sample was washed thoroughly to remove dirt and stain. The sample was placed in the shade for almost 20 days in order to get dry. After drying, the sample was grounded into powder form. An aqueous solution was made of the powder form. The patent was filed, Abbas Nutraceutical Product made from locally available medicinal plant *B. lycium* Royle.

### 2.7. HPLC Analysis of Alkaloids

The quantification of berberine from the root extract of *B. lycium* was carried out by using HPLC, Cat ^#^ PM 951505-0, column C-18 isocratic, 5 *µ*m, 4.6 mm × 250 mm. The liquid chromatography used was DLC-20 by Star-Chrom Lite. The software used was also Star-Chrom. The single-beam UV-spectrophotometer by IRMECO Germany, Model ^#^2020, was used for spectrum analysis and absorbance peak comparison. The mobile phase contains 50 mM potassium dehydrogenase phosphate and acetonitrile in 70 : 30, and pH of solution was adjusted to 3 with phosphoric acid. The flow rate was retained 1 ml/min, and the injection volume was 20 *µ*l. The berberine quantification was done at 271 nm. The peak in the *B. lycium* Royle sample was observed by retention time. The analysis was conducted in triplicate, and berberine was found. The validated method for HPLC is given in [28].

### 2.8. Statistical Analysis

The data in this study were expressed as a mean of triplicate. Statistical comparison and one-way ANOVA followed by Dunnett's multiple comparisons test were made in Prism, version 6.00, GraphPad software for Windows, La Jolla, California, USA, http://www.graphpad.com.

## 3. Results and Discussions

There are 10 districts in Azad Jammu and Kashmir. Data were collected from five districts of AJ&K, i.e., Muzaffarabad, Hattian, Bagh, Poonch, and Neelum, as shown (Table 1). These five districts were selected because they cover the major area of *B. lycium* Royle in the state of AJ&K.

### 3.1. Ethnobotanical Study

In the current study, there were 35 informants (17 males and 18 females) having age ranging from 22 to 75 years. Among them, 11 were housewives, 10 were teachers, 9 were shopkeepers, 3 were farmers, and 2 were lecturers. The information (local name, mode of preparation, and medicinal uses) was collected through questionnaire, interviews, and discussions with villagers. Our questionnaire allowed descriptive response on plant prescribed, plant part used, and detailed information on the mode of preparation (paste, powder, and juice). Root bark powder was used for treating different diseases in the form of paste, given orally or placed on a wound or cut directly (Table 2). Ethnobotany is perhaps the most important method to study natural resources and their interaction by indigenous peoples. Traditional knowledge of these resources, orally transferred from generation to generation, allowed us to work with local people to explore the importance of plant [29]. This study provided information about some therapeutic uses of *B. lycium* Royle. It was found that medicinal values of *B. lycium* Royle are difficult to maintain because of their potential uses; therefore, they are recommended for viable harvest, not being used as fire wood [30]. People use plants in various ways such as medicine, timber wood, fuel wood, food, and fodder [31].

### 3.2. TPC Estimation

TP contents' amount was estimated by using Folin–Ciocâlteu's phenol reagent and is denoted in GAE (Table 3). The highest phenolic contents of roots were observed in Medan Syedan (53.85 ± 1.11 *µ*g/g) and the lowest in Qadrabad (9.50 ± 0.95 *µ*g/g). The phenolic contents of stem showed the highest value of 56.39 *µ*g/g ± 2.01 in Medan Syedan and the lowest value of 8.18 ± 0.72 *µ*g/g. The phenolic contents of leaves were the highest in Patikka (Chanjhal) (88.66 ± 1.07 *µ*g/g) and the lowest in Dhaman Jholi (8.24 ± 1.25 *µ*g/g). The thorn showed the highest concentration of 61.22 ± 1.4 *µ*g/g in Patikka (Chanjhal), and 11.14 ± 1.7 *µ*g/g was the value for Dhaman Jholi. Patikka (Chanjhal) again showed the highest value of phenolic contents in fruits of 66.43 ± 1.09 *µ*g/g, and Dhaman Jholi was the lowest with 10.36 ± 1.47 *µ*g/g. TP contents varied among the plant samples collected from different locations. The variation of phenolic contents was due to environment, soil texture, and altitude differences. It could be said that phenolic content variations were the result of a plant's interaction to its environment. The change in phenols directly affects the medicinal quality of the plant [32]. The main cause for the variation in phenolic contents was due to difference in soil texture, environment, and altitude. Stem, leaf, and inflorescent characters were classified for the identification of *Berberis* species [33].

### 3.3. Estimation of Chlorophyll

Chlorophyll concentrations were calculated in different demographic regions. The values of chlorophyll a and chlorophyll b and the total amount of chlorophyll were expressed as *µ*g/ml (Table 4). The chlorophyll a content was highest (2.16 ± 0.13 *µ*g/ml) in Bagh and lowest (0.24 ± 0.06 *µ*g/ml) in Shahkot. The chlorophyll b was highest in Sathrian (2.66 *µ*g/ml ± 0.41) and lowest in Rawalakot (0.15 ± 0.04 *µ*g/ml). The total chlorophyll content was found highest in Sathrian (3.75 ± 0.53 *µ*g/ml) and lowest in Sheesha Mali (0.53 ± 0.15 *µ*g/ml). The chlorophyll content changed in different areas as well as within the same plant due to differences in leaves' reception of sunlight. It also varied in different areas due to shade and time of exposure to sunlight [20].

### 3.4. DPPH Radical Scavenging Assay

The DPPH method is used for the radical scavenging activity of antioxidants. DPPH is a stable organic free radical and presents the ability to accept hydrogen radical or an electron. Scavenging activity was calculated in percentage of inhibition (Table 5). The IC50 for stem showed the highest value of 810.51 *µ*g/ml in Serli Scha and the lowest for Kaalis (36.63 *µ*g/ml). The IC50 for root showed the highest value of 513.33 in Serli Scha and the lowest for Bakreyali (33.26 *µ*g/ml). The IC50 for leaves showed the highest value of 481.23 *µ*g/ml in Sarran Chatiyan and the lowest for Subhai Mali (40.82 *µ*g/ml). Bakreyali showed 33.26 *µ*g/ml. The IC50 for thorn showed the highest value of 474.14 *µ*g/ml for Laala and the lowest for Bagna (8.69 *µ*g/ml). The highest antioxidant activity was exhibited by the thorn of plants collected from Bagna, having the lowest IC50 of 8.69 *µ*g/ml. Stem and fruits showed the highest antioxidant activity compared with other parts, while roots also exhibited good antioxidant potential. The root bark of *B. lycium* is the best antioxidant compared to ascorbic acid and many other plants [20]. Antioxidant activity among the different parts of the plant and among different plants varies depending on the function and mechanism of phenolic compounds [34]. The antioxidant activity is also due to alkaloids present in its different parts, and that may be a reason that phenolic contents and antioxidant activity are not related very much in the present study [35].

### 3.5. Extraction of Alkaloids from the Root Bark

Berberine is a major alkaloid that is found in *B. lycium* Royle, having a concentration of 4.1% in the root bark of the plant [15]. Berberine shows significant phytotherapeutic benefits [10, 16]. Berberine can be extracted from *B. lycium* Royle roots, fruits, leaves, and stem [9]. Berberine is a major alkaloid present in *Berberis* species and is said to be a very active compound with various pharmacological properties [36]. Berberine is considered as the most important alkaloid, mainly used by the inhabitants to solve health problems [20]. There are two types of alkaloids, namely, palmatine and berberine, extracted from roots of this medicinal plant [37].

### 3.6. Concentration of Berberine

Berberine is a major alkaloid found in our product *B. lycium* Royle, having a concentration of 4.76 percent in root bark as estimated by HPLC (Figure 2).

### 3.7. Syrup Formation and Chemical Composition

Syrup formation was done by adding these constituents, i.e., the root bark extract of *B. lycium* Royle, sorbitol, methylene paraben, propyl paraben, propylene glycerol, dextrose, and flavour. Chemical composition of syrup per serving (1 table spoon): vitamin A (56.75 microgram), vitamin C (1.94 mg), calcium (3.24 mg), sodium (1.68 mg), phosphorous (2.73 mg), potassium (13.1 mg), iron (0.17 mg), zinc (1.88 mg), Mn (0.0055 mg), and berberine (0.95 mg). Fruits and thorns may be used for the development of antioxidant compounds or combinations. Fruits could also be used in its raw form [16]. A wide variety of minerals are also documented in *B. lycium* Royle such as Na, Cu, Ca, S, Fe, Zn, Mn, and Pb that is enough to prepare syrup [15, 16]. Nowadays, nutraceuticals become popular among scientists and are made from medicinal plants [37].

## 4. Conclusion

*Berberis lycium* Royle is under heavy pressure from human activities including overexploitation, overgrazing, deforestation, and unscientific ways of collection. An increase in human population leads to depletion of natural resources. Because of the low potential of natural regeneration, constant high use is posing a great risk to *B. lycium* Royle. Increased livestock is also destroying this plant as they graze its leaves and branches due to its good taste. Goats specifically like to feed on this plant. The increasing human population is destroying the habitat of the plant. Habitat degradation is also due to deforestation, overexploitation, livestock grazing, and unscientific ways of collection. Other factors contributing to this problem are fuel wood cutting, stall feeding, soil erosion, fires, lack of awareness, weak law enforcement, and smuggling. As root bark of *B. lycium* Royle is used for the treatment, local Hakeems are using every possible way to obtain roots, resulting damage to the population of *B. lycium* Royle. Because of lack of awareness, people use this plant for stall feeding their animals and fire fuel, so in recent years, it has been vanished from a big area. It is the need of the hour to take the immediate attention to conserve this species.

The TPC was high in leaf samples collected from Chanjhal, Muzaffarabad District of AJ&K. The highest total chlorophyll contents were found in samples collected from Sathrian, Neelum District. The highest antioxidant activity with the lowest IC50 values was obtained from the root sample collected from Bakreyali, Muzaffarabad District, as compared with other districts. The concentration of berberine was found to be 4.76 percent in the root bark (sample collected from Muzaffarabad District) of *B. lycium* Royle, estimated by high-performance liquid chromatography (HPLC). In syrup composition, 0.95 mg/5 ml of berberine was used. *B. lycium* Royle possesses powerful antioxidant activity in its all parts, especially root, stem, and fruit. Fruits are already used as food in hilly areas of AJ&K. Another important finding from the present study is that change in the environment has a big impact on the chemical composition of the same species, so its medicinal properties get changed. Hence, it is concluded that amongst the five districts, the plant parts (stem, fruits, and root) collected from Muzaffarabad District, AJ&K, showed the highest medicinal potential due to its unique climatic conditions.

## Figures and Tables

**Figure 1:** District-wise map of Azad Jammu and Kashmir; the districts from which samples were collected in the current study are labeled with red-colored star.

**Figure 2:** The retention peak of HPLC in berberine reference (a). The retention peak of *B. lycium* Royle sample collected from Patikka, Muzaffarabad, AJ&K (b).

**Table 1:** Information of five districts of AJ&K from where *B. lycium* Royle samples were collected.

District	Altitude (feet)	Latitude (°N)	Longitude (°E)	Flowering season	Fruit ripening season
Muzaffarabad	58147	34.38362	73.471054	April-May	June–August
Hattian	5362.167	34.26704	73.7432	April-May	June–August
Bagh	2107.5	33.9441151	73.7918	April–June	July–October
Poonch	5051.5	33.8423496	73.7507	June-July	August–October
Neelum	14989.5	34.49522	73.9106	April-May	July-August

Local name of the plant is “sunbal.”

**Table 2:** The number of informants who have used *B. lycium* Royle to treat different diseases.

S. no.	Root bark powder used for treating different diseases	No. of informants
1	Joint pain	3
2	Diarrhea and joint pain	2
3	Diabetes and joint pain	2
4	Diabetes	4
5	Broken bone and arthritis	6
6	Broken bones	16
7	Arthritis	2
	Grand total	35

**Table 3:** Total phenolic contents estimated in root, stem, leaves, thorn, and fruits of *Berberis lycium* Royle.

Source/location	Total phenolic contents				
	Root (*µ*g/g ± SD)	Stem (*µ*g/g ± SD)	Leaves (*µ*g/g ± SD)	Thorn (*µ*g/g ± SD)	Fruit (*µ*g/g ± SD)
Serli Scha	16.77 ± 0.89	14.60 ± 0.72	35.74 ± 1.10	23.90 ± 1.89	25.46 ± 0.77
Copra Gali	18.50 ± 0.66	23.45 ± 0.92	17.69 ± 0.87	21.53 ± 2.04	18.67 ± 0.67
Sadbun	9.56 ± 1.02	10.45 ± 0.58	13.56 ± 1.27	12.57 ± 1.90	11.52 ± 1.11
Patikka (Chanjhal)	50.16 ± 1.78	42.75 ± 0.90	88.66 ± 1.07	61.22 ± 1.45	66.43 ± 1.09
Bakreyali	12.08 ± 1.65	43.27 ± 0.71	38.71 ± 0.79	34.02 ± 2.57	28.66 ± 1.47
Ranjhata	15.80 ± 1.11	22.44 ± 0.92	33.47 ± 1.31	24.10 ± 1.10	24.75 ± 0.47
Garhi Dupatta	12.33 ± 1.57	8.18 ± 0.72	12.11 ± 1.82	12.49 ± 2.30	12.05 ± 1.58
Dhaman Jholi	12.40 ± 1.78	10.19 ± 0.70	8.24 ± 1.25	11.14 ± 1.73	10.36 ± 1.47
Bagh	12.18 ± 1.88	10.45 ± 0.87	14.35 ± 2.22	12.12 ± 1.02	12.55 ± 1.36
Arja	45.77 ± 1.17	14.27 ± 1.00	31.80 ± 2.81	30.97 ± 1.49	35.71 ± 1.28
Qadrabad	9.50 ± 0.95	44.72 ± 1.11	12.23 ± 1.62	22.91 ± 1.59	14.67 ± 1.26
Rawalakot	18.62 ± 1.44	33.69 ± 1.31	31.20 ± 1.64	28.05 ± 1.41	25.40 ± 0.94
Khrick	27.12 ± 1.50	33.39 ± 0.90	19.55 ± 1.08	27.00 ± 1.51	24.54 ± 1.34
Bhanjhosa	15.85 ± 1.15	23.37 ± 1.18	34.38 ± 2.00	24.17 ± 1.18	24.34 ± 0.97
Haryala	13.59 ± 1.31	11.56 ± 1.02	11.75 ± 2.23	12.71 ± 1.90	12.40 ± 1.57
Subai Mali	37.88 ± 1.05	24.38 ± 1.01	10.41 ± 2.12	25.04 ± 1.44	24.21 ± 1.18
Sheesha Mali	15.80 ± 0.92	14.53 ± 1.26	10.80 ± 1.95	13.25 ± 1.05	12.81 ± 0.95
Kalis	12.52 ± 1.37	11.25 ± 0.81	11.49 ± 3.01	11.45 ± 1.75	10.58 ± 1.10
Sarran Chatiyan	10.59 ± 1.01	10.53 ± 1.02	12.71 ± 1.94	12.14 ± 2.77	11.32 ± 1.27
Gori Syedan	13.19 ± 0.93	13.28 ± 1.18	12.09 ± 1.36	14.01 ± 2.34	11.95 ± 0.50
Neelum	9.53 ± 1.38	22.42 ± 1.99	34.40 ± 0.83	23.67 ± 2.68	22.42 ± 1.57
Ziarat	14.26 ± 0.73	19.43 ± 1.29	12.82 ± 0.79	16.05 ± 1.43	14.66 ± 1.24
Thanger	14.88 ± 1.17	19.36 ± 1.50	17.47 ± 0.65	17.27 ± 1.13	16.26 ± 0.69
Chinar Pura	12.67 ± 0.81	13.49 ± 1.19	11.68 ± 1.98	12.86 ± 1.58	11.67 ± 1.16
Shahkot	13.46 ± 1.16	14.04 ± 1.69	10.99 ± 1.48	12.89 ± 1.54	12.16 ± 1.17
Bagna	16.65 ± 1.48	15.13 ± 1.24	14.30 ± 0.98	15.83 ± 1.64	14.57 ± 0.62
Medan Syedan	53.85 ± 1.11	56.39 ± 2.01	13.24 ± 1.08	41.33 ± 0.96	35.68 ± 0.95
Lawat	18.77 ± 1.21	16.24 ± 1.61	17.41 ± 0.82	17.56 ± 0.78	17.73 ± 1.05
Kundal Shahi	13.56 ± 1.42	13.72 ± 1.92	31.47 ± 0.65	19.40 ± 1.08	21.87 ± 1.46
Sathrian	34.89 ± 1.13	27.75 ± 1.89	46.95 ± 1.54	36.83 ± 1.08	40.12 ± 1.81
Laala	15.40 ± 0.64	13.92 ± 1.60	11.23 ± 2.47	13.92 ± 1.61	12.63 ± 0.74
Palang	18.23 ± 0.71	15.10 ± 1.37	13.09 ± 1.31	15.38 ± 0.96	15.46 ± 0.79
Keran	16.47 ± 1.08	12.23 ± 1.87	12.53 ± 2.23	13.50 ± 1.77	13.34 ± 1.01
Ethai	13.29 ± 0.83	12.74 ± 2.18	13.11 ± 1.26	13.53 ± 2.05	13.15 ± 1.22
Slam Pura	22.19 ± 1.26	13.28 ± 1.43	9.13 ± 1.19	14.54 ± 1.11	15.97 ± 1.76

The *P* value was <0.0001, and the CI was 99 percent.

**Table 4:** Chlorophyll a, chlorophyll b, and total chlorophyll in *B. lycium* Royle of different places having a variety of chlorophyll contents due to differences in the environment of places.

Location of the samples	Chlorophyll a (*µ*g/ml ± SD)	Chlorophyll b (*µ*g/ml ± SD)	Total chlorophyll (*µ*g/ml ± SD)
Serli Scha	1.52 ± 0.35	0.27 ± 0.07	1.79 ± 0.41
Copra Gali	1.69 ± 0.09	0.31 ± 0.07	2.01 ± 0.05
Sadbun	1.21 ± 0.20	1.03 ± 0.09	2.24 ± 0.28
Patikka (Chanjhal)	0.96 ± 0.16	1.31 ± 0.20	2.27 ± 0.18
Bakreyali	1.12 ± 0.06	1.11 ± 0.16	2.23 ± 0.16
Garhi Dupatta	0.33 ± 0.10	1.32 ± 0.26	1.65 ± 0.17
Dhaman Jholi	1.29 ± 0.23	2.42 ± 0.18	3.71 ± 0.15
Bagh	2.16 ± 0.13	1.41 ± 0.04	3.57 ± 0.09
Arja	1.41 ± 0.14	0.23 ± 0.05	1.65 ± 0.09
Qadrabad	0.53 ± 0.07	0.69 ± 0.07	1.23 ± 0.14
Rawalakot	1.47 ± 0.13	0.15 ± 0.04	1.62 ± 0.12
Khrick	1.49 ± 0.20	0.24 ± 0.04	1.73 ± 0.20
Bhanjhosa	1.52 ± 0.17	0.40 ± 0.02	1.92 ± 0.15
Haryala	0.28 ± 0.06	0.70 ± 0.11	0.98 ± 0.16
Subai Mali	0.49 ± 0.09	2.45 ± 0.08	2.94 ± 0.14
Sheesha Mali	0.26 ± 0.02	0.30 ± 0.14	0.56 ± 0.15
Kalis	0.64 ± 0.15	0.71 ± 0.09	1.35 ± 0.21
Sarran Chatiyan	0.53 ± 0.18	1.42 ± 0.27	1.95 ± 0.12
Gori Syedan	1.51 ± 0.14	0.66 ± 0.15	2.17 ± 0.06
Neelum	0.92 ± 0.09	0.79 ± 0.19	1.71 ± 0.20
Ziarat	1.90 ± 0.07	0.77 ± 0.10	2.67 ± 0.03
Thanger	1.72 ± 0.22	0.37 ± 0.12	2.09 ± 0.31
Chinar Pura	0.97 ± 0.06	1.21 ± 0.23	2.18 ± 0.18
Shahkot	0.24 ± 0.06	0.41 ± 0.05	0.65 ± 0.07
Bagna	0.67 ± 0.09	1.72 ± 0.28	2.39 ± 0.36
Medan Syedan	0.94 ± 0.16	0.84 ± 0.01	1.78 ± 0.17
Lawat	0.55 ± 0.08	1.72 ± 0.27	2.26 ± 0.28
Kundal Shahi	0.66 ± 0.14	1.16 ± 0.11	1.82 ± 0.11
Sathrian	1.10 ± 0.12	2.66 ± 0.41	3.75 ± 0.53
Laala	0.60 ± 0.19	1.39 ± 0.40	1.99 ± 0.60
Palang	1.41 ± 0.19	0.17 ± 0.07	1.57 ± 0.13
Keran	0.26 ± 0.14	1.48 ± 0.16	1.74 ± 0.07
Ethai	1.35 ± 0.33	1.38 ± 0.45	2.73 ± 0.34
Slam Pura	1.60 ± 0.17	1.65 ± 0.20	3.24 ± 0.31

*P* value <0.0001 and CI = 99%.

**Table 5:** IC50 concentrations in *B. lycium* Royle.

Source	DPPH IC50 of *B. lycium* Royle				
	Root	Stem	Leaves	Thorn	Fruit
Serli Scha	513.33	810.52	150.89	43.94	662.24
Copra Gali	103.97	586.16	132.24	343.16	382.51
Sadbun	501.38	154.19	168.48	163.24	463.95
Patikka (Chanjhal)	122.72	39.54	382.72	70.21	340.50
Bakreyali	33.26	211.98	123.32	215.08	409.37
Ranjhata	190.54	157.67	150.80	355.34	154.84
Garhi Dupatta	244.44	469.71	457.84	444.47	411.55
Dhaman Jholi	218.57	231.64	136.00	76.25	217.98
Bagh	176.59	397.57	391.96	443.50	162.13
Arja	219.24	471.85	40.83	167.38	169.37
Qadrabad	466.86	406.33	236.74	183.62	202.42
Rawalakot	401.07	36.64	207.59	280.19	368.04
Khrick	206.74	178.47	481.23	455.59	435.09
Bhanjhosa	149.25	472.25	153.68	47.44	368.04
Haryala	375.42	376.13	433.84	239.11	461.68
Subai Mali	406.80	335.92	200.92	154.16	418.66
Sheesha Mali	183.62	215.41	330.19	177.40	398.18
Kalis	141.83	390.21	448.05	418.28	273.43
Sarran Chatiyan	163.17	417.94	170.57	440.38	119.02
Gori Syedan	384.60	141.73	399.00	203.39	468.88
Neelum	221.07	457.58	194.63	74.48	469.26
Ziarat	152.34	447.73	182.89	46.07	177.60
Thanger	256.81	199.24	219.52	270.24	234.79
Chinar Pura	113.04	225.69	458.56	202.94	73.16
Shahkot	253.37	128.21	372.11	87.46	374.93
Bagna	411.86	477.51	362.20	8.70	360.01
Medan Syedan	252.29	130.99	243.34	342.59	438.27
Lawat	167.40	307.55	173.40	203.19	31.01
Kundal Shahi	382.77	423.19	295.02	456.71	74.40
Sathrian	138.77	333.25	191.60	226.68	371.96
Laala	143.82	315.15	437.53	474.15	468.42
Palang	47.06	392.23	261.11	196.18	147.96
Keran	378.59	39.18	202.14	245.97	226.53
Ethai	103.08	423.16	211.22	257.16	163.53
Slam Pura	513.33	810.52	150.89	43.94	662.24

IC50 is the concentration at which 50% scavenging activity is inhibited.

## Data Availability

The data used to support the findings of this study are included within the article.
